# Clinical Efficacy of Tacrolimus Ointment + 3% Boric Acid Lotion Joint Chinese Angelica Decoction in Chronic Perianal Eczema

**DOI:** 10.1155/2021/1016108

**Published:** 2021-10-21

**Authors:** Weiwei Gao, Xueli Qiao, Jinxin Zhu, Xin Jin, Yuegang Wei

**Affiliations:** ^1^The First Clinical Medical College of Nanjing University of Chinese Medicine, Nanjing, Jiangsu 210023, China; ^2^Department of Proctology, Affiliated Hospital of Xuzhou Medical University, Xuzhou, Jiangsu 221004, China; ^3^Department of Pharmacy, The Affiliated Huai'an Hospital of Xuzhou Medical University, Huai'an Second People's Hospital, Huai'an, Jiangsu 223002, China; ^4^Science and Education, Lianshui County People's Hospital, Huai'an 223400, China; ^5^Dermatology Department of Affiliated Hospital of Xuzhou Medical University, Xuzhou 221004, China

## Abstract

**Objective:**

To unearth the clinical efficacy of tacrolimus ointment + 3% boric acid lotion joint Chinese angelica decoction in chronic perianal eczema.

**Methods:**

Patients with chronic perianal eczema admitted to hospital from June 2018 and June 2019 were retrospectively analyzed. Patients in the control group (*n* = 38) underwent basic therapy with tacrolimus ointment + 3% boric acid lotion, whereas those in the observation group (*n* = 38) were given oral Chinese angelica decoction on the basis of the above therapy. Patient's baseline information before therapy and clinical symptoms after therapy were observed and compared, including pruritus ani score, anus drainage and damp score, skin lesion score, skin lesion area score, life quality index score, and IL-2, IL-4, and IgE levels in serum. Overall efficacy in the two groups was also evaluated.

**Results:**

No significant differences were found in the baseline information between the observation group and control group before therapy. After therapy, pruritus ani score (*P* = 0.023), anus drainage and damp score (*P* = 0.041), skin lesion score (*P* = 0.025), and skin lesion area score (*P* = 0.035) of patients in the observation group were remarkably lower than those in the control group. Significantly higher release levels of clinical symptoms of patients in the observation group were indicated. With respect to the control group, the life quality score (*P* = 0.020) and IgE level in serum (*P* = 0.003) of patients in the observation group were significantly lower, while IL-4 level in serum was significantly higher (*P* = 0.129). The therapy in the observation group achieved better clinical efficacy. Overall efficacy in the observation group was markedly favorable with respect to the control group.

**Conclusion:**

With respect to tacrolimus ointment + 3% boric acid lotion, patients with chronic perianal eczema displayed better clinical efficacy after jointly being treated by Chinese angelica decoction.

## 1. Introduction

Perianal eczema is a skin disease in perianal skins and mucosae and may spread to perineal region and externalia [1]. Clinical symptoms of perianal eczema are pruritus, calor, and exudative lesions. Three main types like irritant toxic, atopic, and anaphylactic contact dermatitis may be caused by various colon diseases, skin diseases, anaphylactic diseases, or pathogens [2–4]. To date, glucocorticoid drugs are given to treat perianal eczema patients and can achieve relatively ideal efficacy in the early stage. However, a massive number of investigations suggested that patients are prone to rely on these drugs, and after withdrawal, they are prone to suffer from disease recurrence and adverse events [5, 6]. A more effective alternative is therefore urgent for disease treatment.

With the emergency and application of topical calcineurin inhibitors for perianal eczema treatment, their anti-inflammatory, immunoregulation, and steroid retention functions attract much attention. The nonsteroidal anti-inflammatory drugs (pimecrolimus and tacrolimus) display favorable efficacy in treating assertive perianal eczema [7–9]. Nonetheless, relevant investigations are still lacking. In addition, boric acid lotion can also be used for perianal eczema. Bai et al. [10] also revealed the suppression of boric acid lotion on bacteria and fungi. Currently, the extensively used treatment for perianal eczema is boric acid lotion plus tacrolimus ointment [6].

Traditional Chinese medicines (angelica sinensis and radix sophorae flavescentis) are beneficial to treatment for eczema [11, 12]. Thus, we speculated that it is meaningful to apply Chinese angelica to the treatment of perianal eczema. Joint treatment of Chinese and Western medicine may achieve unanticipated clinical benefits. Chinese angelica decoction originates from the Sixth Chapter of Yan's Prescription for Rescuing Lives (Jishengfangjuan VI): Chinese angelica decoction is mainly used for retention of qi and blood, internal wind-heat, symptoms like scabies, swelling, itch, pus, or reddish measles. It is composed of 50 g of Chinese angelica (remove residual stems, leaf stems, and rhizomes), white peony, Ligusticum wallichii, Rehmannia glutinosa (washed), Tribulusterrester (fried; remove shoots), Saposhnikovia divaricate (remove residual stems, leaf stems, and rhizomes), and Schizonepeta tenusfolia Briq, and 25 g of Fallopia multiflora (Thunb.) Harald, Astragalus mongholicus Bunge (remove residual stems, leaf stems, rhizomes), and Glycyrrhiza uralensis (baked). Major efficacies of this drug are replenishing qi and blood, treating skin diseases whose overall pathogeneses are blood dryness and wind-heat including scabies, urticaria, skin pruritus, feet and hands chap, withered appearance, and stubborn ringworm [13]. Chinese angelica decoction is a classical prescription for skin inflammation. A preceding investigation discovered the favorable benefit of Chinese angelica decoction in treating chronic perianal eczema, which is worth being introduced [14]. The clinical efficacy of Chinese angelica decoction joint tacrolimus ointment + 3% boric acid lotion has been rarely involved.

This investigation systematically researched tacrolimus ointment + 3% boric acid lotion joint Chinese angelica decoction on chronic perianal eczema. Patients in the control group (*n* = 38) underwent basic therapy with tacrolimus ointment + 3% boric acid lotion, whereas those in the observation group (*n* = 38) were given Chinese angelica decoction on the basis of the above therapy.

## 2. Methods

### 2.1. Sample Collection and Grouping

Totally, 76 perianal eczema patients were included as research objects. Diagnosis criteria were rough and hypertrophic perianal skin, lichenification, accompanied hyperpigmentation, symmetrically distributed and frequently recurrent rash, and itchy or extremely itchy. All patients were diagnosed and systematically treated in hospital during June 2018-June 2019. They were divided into a control group (*n* = 38) and an observation group (*n* = 38) according to therapy plans. No significant differences were found in the baseline information of perianal eczema patients in two groups (see Table 1).

### 2.2. Treatment Plans

Two groups of patients were hydropathic compressed with 3% boric acid lotion (Shanghai Yunjia Huangpu Pharmaceutical Co., Ltd.; State Medical Permitment No. H31022883) and then smeared with tacrolimus ointment (LEO Laboratories Ltd.; active ingredient: 3 mg/10 g; Registration No. HJ20181015) in perianal region. The overall treatment cycle includes 2 courses; 2 weeks a course; twice a day. In addition, the observation group was given Chinese angelica decoction orally for 2 weeks a course for 2 courses. Chinese angelica decoction contains 15 g angelica, 30 g Rehmannia glutinosa, 20 g radix paeoniae alba, 10 g ligusticum chuanxiong hort, 15 g polygonum multiflorum, tenuifolia, 10 g saposhniovia root, 20 g tribulusterrestris, 30 g astragalus membranaceus, and 6 g licorice roots (one dose orally every day).

### 2.3. Observation Criteria

#### 2.3.1. Pruritus Ani Score before and after Treatment

Visual analogue scale (VAS) was adopted to assess pruritus ani before and after treatment [15]. To be specific, 10 cm VAS was divided into 0-10.0 for no pruritus ani, 10 for intense pruritus ani and unable to sleep, and middle numbers for different levels of pruritus ani. Patients were instructed to correspond their pruritus ani to a specific location of the scale and physicians scored them on this basis.

#### 2.3.2. Anus Drainage and Damp Score [16] before and after Treatment

0 point: no seepage; 1 point: a little seepage (occasionally moist); 2 points: plenty of seepage (evident perianal maceration); 3 points: a great amount of seepage (perianal maceration pollutes underwear).

#### 2.3.3. Skin Lesion Score [17] before and after Treatment

Papule: 1 point-mild (slight red, scattered distribution, and no phlysis); 2 points-moderate (reddish, close distribution, and visible papulovesicle); 3 points-severe (rather red, very close distribution, and scattered phlysis). Erosion: 0 point-no erosion; 1 point-mild erosion (scattered distribution); 2 points-moderate erosion (small spots and partly confluent); 3 points-severe erosion (evident and vast erosion). Effusion: 0 point-no effusion; 1 point-mild effusion (scattered distribution and hard to observe); 2 points-mild effusion (much effusion and easily to soak toilet paper); 3 points-severe effusion (very much effusion and in the shape of beads).

#### 2.3.4. Skin Lesion Area Score [18]

Disinfected projection film was used to record the size of the wound on cardiogram paper. Wound area was recorded as the product of the length of the horizontal and vertical axes in cardiogram paper. 0 point-no skin lesion area: 0; 2 points-mild: <2∗2 cm; 4 points-mild: >2∗2 cm and<6∗6 cm; 6 points-severe: >6∗6 cm.

#### 2.3.5. Life Quality Index Score before and after Treatment

Skin disease life quality index was applied to assess changes in life quality [19]. There were 10 questions, each of which was scored by 4-level scoring method: 0, 1, 2, and 3 points. Total score ranges from 0 to 30 points. Higher scores indicate more effects of the disease on patient's life quality.

#### 2.3.6. Overall Efficacy Evaluation Criteria [20]

Referring to Chinese Medicine Clinical Research of New Drugs Guiding Principles, improvement rate of clinical symptom score = (total score of symptom score before treatment–total score of symptom score after treatment)/total score before treatment × 100%. Cure: descend range of symptom score ≥ 90%; very effective: descend range of symptom score ≥ 60% and <90%; effective: descend range of symptom score ≥ 20% and<60%; ineffective: descend range of symptom score < 20%.

#### 2.3.7. Detection of Immune Reaction-Related Proteins

Patient's peripheral blood was drawn before and after treatment to test levels of IL-2, IL-4, and IgE in serum. Changes in the expression levels of the above proteins were observed.

### 2.4. Data Analysis

Data were analyzed by SPSS 26.0 software. Enumeration data were denoted in the form of *n*. Fisher exact test or Chi-square test was used. Measurement data were subjected to tests for normality and homogeneity of variance. Data conforming to normal distribution were displayed by mean ± standard deviation. Differences between data were examined by *t*-test. *P* < 0.05 symbolized statistically significant.

## 3. Results

### 3.1. The Impact of Joint Chinese Angelica Decoction on Clinical Symptom Score of Chronic Perianal Eczema

In this section, we compared several clinical symptom scores of chronic perianal eczema patients after treatment in two groups, including pruritus ani score, anus drainage and damp score, skin lesion score, and skin lesion area score. Scores of two groups of patients both dropped, wherein patient's pruritus ani score (*P* = 0.023), anus drainage and damp score (*P* = 0.041), skin lesion score (*P* = 0.025), and skin lesion area score (*P* = 0.035) in the observation group were significantly lower (Table 2).

### 3.2. The Impact of Joint Chinese Angelica Decoction on Patient's Life Quality Score and Immune Reaction-Related Proteins

In this section, we mainly compared life quality indexes and levels of IL-2, IL-4, and IgE in serum of two groups of patients after treatment. It was found that life quality index score in the observation group was significantly lower (*P* = 0.020) (Figure 1(a)). With respect to the control group, patients in the observation group had lower IL-2 (no significant difference, *P* = 0.129) and IgE (statistical significance, *P* = 0.013) levels and significantly higher IL-4 level (*P* = 0.003) (Figures 1(b)–1(d)).

### 3.3. The Impacts of Tacrolimus Ointment + 3% Boric Acid Lotion Joint Chinese Angelica Decoction on the Overall Efficacy on Patients with Chronic Perianal Eczema

In this section, we compared overall efficacy of two groups of therapy plans. As shown in Table 3, the overall efficacy of patients in the observation group was better than that in the control group (*P* = 0.033).

## 4. Discussion

The purpose of therapy for perianal eczema is to improve patient's clinical symptoms and reduce the impact on patient's life quality [21]. This investigation comprehensively assessed the clinical efficacy of Chinese angelica decoction joint tacrolimus ointment + 3% boric acid lotion on chronic perianal eczema patient's clinical symptom-related indexes, life quality index score, expression changes of immune reaction-related protein level, and overall efficacy.

A compelling investigation described that Chinese angelica decoction joint tacrolimus qu ointment + 3% boric acid lotion can improve T lymphocytes subsets level and reduce skin lesion area and itching level of patients with blood deficiency and dryness type eczema [22]. This investigation enrolled 76 patients with chronic perianal eczema and divided them into the control group and observation group. Changes of each index and overall efficacy of two groups of patients were compared to observe clinical value of Chinese angelica decoction. It was indicated that after two courses of treatment, patients displayed differences in clinical symptom score, life quality score, and clinical efficacy. First, their clinical symptoms were all improved after treatment. Next, the observation group presented favorable therapeutic efficacy in scores of each index and overall efficacy, suggestive of more ideal effect of angelica based on basic therapy. Taken together, tacrolimus ointment + 3% boric acid lotion joint Chinese angelica decoction was more effective than pure basic therapy. Patient's pruritus ani score, anus drainage and damp score, skin lesion score, skin lesion area score, life quality index score and IL-4 and IgE levels in serum, and overall efficacy of treatment were all significantly enhanced.

A preceding investigation elaborated that the absence of AQP3 correlates with intercellular edema and water homeostasis [23]. In the acute or subacute stages of edema, the expression of AQP3 is abnormally reduced in plasma membrane. Increasing the expression of AQP3 in local lesions may inhibit eczema inflammation. Chinese angelica decoction has been proved to strengthen AQP3 gene and protein expressions in the guinea pig psoriasis model [24]. Thus, we posited that a combination of Chinese angelica decoction can enhance perianal eczema treatment, and this impact may be associated with AQP3 regulation. Incremental experiments are planned in the future.

All in all, this investigation verified the clinical efficacy of Chinese angelica decoction joint tacrolimus ointment + 3% boric acid lotion on chronic perianal eczema. The following treatment may take this Chinese and Western medicine combination as a new direction. Limitations shall be considered here. We did not clarify molecular mechanism of Chinese angelica decoction affecting perianal eczema, and clinical samples were not enough. We are about to design experiments to probe the mechanism and supplement recurrence rate-related studies.

## Figures and Tables

**Figure 1:** Life quality index score and laboratory detection index of patients in two groups after treatment. (a) Life quality index score of patients in the observation and control groups after treatment. (b)–(d) IL-2, IL-4, and IgE levels in serum of two groups of patients after treatment, respectively.

**Table 1:** Baseline information of patients in two groups.

Baseline information	Observation group (*n* = 38)	Control group (*n* = 38)	*P* value
Age (years)	41.08 ± 9.05	44.44 ± 11.67	0.262^a^
Course of disease (month)	21.27 ± 10.20	21.43 ± 8.26	0.934^a^
Sex			
Male	15	17	0.817^b^
Female	23	21	
Pruritus ani score	3.76 ± 0.78	4.00 ± 0.52	0.068^a^
Anus drainage and damp score			
1	7	9	0.563
2	12	8	
3	19	21	
Skin lesion score			
0 ~ 3	5	6	0.995
4 ~ 6	20	19	
7 ~ 9	13	13	
Skin lesion area score			
2	5	4	0.882
4	18	20	
6	15	14	
Life quality index score			
0 ~ 10	8	7	0.194
11~20	27	23	
21~30	3	8	
IL-2	65.75 ± 28.48	71.53 ± 23.73	0.386^a^
IL-4	21.31 ± 6.82	20.54 ± 7.57	0.827^a^
IgE	53.01 ± 16.72	51.89 ± 15.58	0.983^a^

Notes: ^a^independent sample *t*-test; ^b^Fisher exact test; all tests were two-tail *P* value.

**Table 2:** Comparison of each clinical symptom score of two groups of patients after treatment.

Clinical symptom score	Observation group (*n* = 38)	Control group (*n* = 38)	*P* value
Pruritus ani score	2.82 ± 0.55	3.10 ± 0.39	0.023^a^
Anus drainage and damp score			
0	10	5	0.041
1	14	8	
2	14	25	
Skin lesion score			
0 ~ 3	28	25	0.025
4 ~ 6	10	13	
Skin lesion area score			
0	11	3	0.035
2	19	20	
4	8	15	

Notes: ^a^independent sample *t*-test; two-tailed *P* value was applied for all tests.

**Table 3:** Comparison of overall efficacy of two groups of patients.

Overall efficacy	Cured	Slightly effective	Effective	In-effective	*P* value
Control group (*n* = 38)	8	9	12	9	0.033
Observation group (*n* = 38)	18	9	9	2	

## Data Availability

The data and materials in the current study are available from the corresponding author on reasonable request.
